The article "Relationship between the Degree of Illness in Elderly Patients with Rheumatoid Arthritis and Parameters of Musculoskeletal Ultrasound and Oswestry Dysfunction Index and Clinical Value Analysis" was retracted in 2023. Reasons: signs of a paper mill; compromised peer review; unreliable results or conclusions.

# Relationship between the Degree of Illness in Elderly Patients with Rheumatoid Arthritis and Parameters of Musculoskeletal Ultrasound and Oswestry Dysfunction Index and Clinical Value Analysis

**DOI:** 10.1155/2022/4307864

**Published:** 2022-08-02

**Authors:** Danping Shen, Zun Li, Zhe Shan, Jue Wang, Yujie Ren

**Affiliations:** ^1^Department of Ultrasound, Wujin Hospital Affiliated with Jiangsu University, Changzhou 213000, Jiangsu, China; ^2^The Wujin Clinical College of Xuzhou Medical University, Changzhou 213000, Jiangsu, China; ^3^Department of Blood Rheumatism, Wujin Hospital Affiliated with Jiangsu University, Changzhou 213000, Jiangsu, China

## Abstract

**Objective:**

The aim of the study is to explore the relationship between the degree of illness in elderly patients with rheumatoid arthritis (RA) and parameters of musculoskeletal ultrasound (MSUS) and Oswestry Dysfunction Index (ODI) and its clinical value.

**Methods:**

The clinical data of 100 elderly patients with RA admitted to our hospital from May 2016 to May 2022 were retrospectively analyzed. The patients were divided into four groups, including the remission group (DAS28 ≤ 2.6, *n* = 25), low activity group (2.6 ≤ DAS28 ≤ 3.2, *n* = 25), middle activity group (3.2 ≤ DAS28 ≤ 5.1, *n* = 25), and high activity group (DAS > 5.1, *n* = 25) according to the disease activity score-28 (DAS28). All patients underwent ultrasonic detection to compare the relationship between the degree of illness in elderly patients with RA and parameters of MSUS and ODI.

**Results:**

The total semiquantitative score of MSUS and ODI score in the remission group were obviously lower than those in the other three groups (*P* < 0.001). The degree of illness in elderly patients with RA was positively correlated with parameters of MSUS (*r* = 0.886, *P* < 0.001). The degree of illness in elderly patients with RA was positively correlated with ODI (*r* = 0.907, *P* < 0.001).

**Conclusion:**

The degree of illness in elderly patients with RA is closely related to parameters of MSUS and ODI, and the parameters of MSUS have a higher evaluation value for the degree of illness in elderly patients with RA, which are correlated with ODI.

## 1. Introduction

As a common disease in the rheumatic immunology department, rheumatoid arthritis (RA) is a chronic and systemic autoimmune disease, with aggressive and symmetric polyarthritis as the main clinical manifestations [1], and its clinical symptoms are limb fatigue, muscle soreness in the whole body, and joint swelling. At present, the complex etiology and pathogenesis of RA have not been fully elucidated, which may be related to microbial infection, smoking, and autoimmunity, and heterogeneity exists even in the same type, with different etiology in various types [2]. Furthermore, the disease often involves the small joints of extremities like hands and feet, which seriously affects the joint function and daily life in the late stage, and even loses the self-care ability. In addition, the adverse factors such as toxicity and side effects and economic pressure in the treatment process cause great pressure on the patient's body and mind, resulting in a significant decline in quality of life [3]. According to relevant literature, the incidence of RA is the highest in systemic connective tissue disease mostly in women aged 35–55 years old, with the incidence as 0.49%, and the incidence and disability rate of RA increase with age [4]. According to statistics, the number of patients with RA accounts for about 0.99% of the global population, with the prevalence rate in China at about 0.29%, and the ratio of male to female morbidity is about 1 : 2.4 [5]. Skielta Mattias et al. [6] have noted that the 4–9 years of mutilation rate is about 59.99% if RA patients do not receive timely treatment, and the disability rate over 25 years is 89.99%, which seriously affects the health of patients.

Wang Qiyu et al. [7] have pointed out that early diagnosis of RA, assessment of disease activity, and analysis of ODI are the key to treatment selection and prognosis improvement. Radiological imaging is a common clinical diagnosis and treatment method, but this method is expensive and has a radioactive injury, which is not easily accepted by patients [8, 9]. However, characterized by no radiation, no wound, and convenient operation, musculoskeletal ultrasound (MSUS) has been widely used in the early diagnosis of RA, but there are also shortcomings in this diagnostic technique, for example, the examination results are easily affected by the operatives, and the lesions in the large joint cannot be effectively examined. Zhang Shibin et al. [10] have found that the degree of illness in patients is associated with a semiquantitative score of MSUS. At the same time, the scale of the Oswestry Disability Index (ODI) was designed by Fairbank and other experts in 1976. After a large number of trial questionnaires, version 1.0 of ODI was formed in 1980, which was widely promoted at the Paris International Conference on Studies of Lumbar Vertebra, and the evaluation of the ODI scale adopted in elderly patients with RA can directly reflect the degree of illness [11]. It has been confirmed that the ODI scale, as a measurement instrument for functional impairment, has good reliability and validity in chronic low back pain and lumbar disc herniation [12]. However, there are few reports on the relationship between the degree of illness in elderly patients with RA and parameters of MSUS and ODI and clinical value. Based on this, this study adopted the scheme and carried out the joint clinical intervention on subjects in order to provide more clinical evidence-based proof for such patients.

## 2. Materials and Methods

### 2.1. General Information

The clinical data of 100 elderly patients with RA admitted to our hospital from May 2016 to May 2022 were retrospectively analyzed. The patients were divided into four groups, including the remission group (DAS28 ≤ 2.6, *n* = 25), low activity group (2.6 ≤ DAS28 ≤ 3.2, *n* = 25), middle activity group (3.2 ≤ DAS28 ≤ 5.1, *n* = 25), and high activity group (DAS > 5.1, *n* = 25) according to the disease activity score-28 (DAS28). This study was consistent with the Declaration of Helsinki (2013) [13].

### 2.2. Recruitment of Study Subjects

#### 2.2.1. Inclusion Criteria

The inclusion criteria were as follows: (1) those who met the diagnostic criteria of RA in the Chinese Guidelines for the Diagnosis and Treatment of Rheumatoid Arthritis 2018 [14] and were diagnosed with RA by clinic and imaging examinations, with the manifestations of clinical symptoms as muscle soreness in the whole body, articular pain, and appetite depression. (2) Those who had symptoms like varying degrees of joint swelling, pain, and activity limitation. (3) Those who were above the age of 18, without the limitation of gender. (4) Those who did not take the related drugs such as anti-infective drugs or glucocorticoids affecting the study results within three months before joining the group.

#### 2.2.2. Exclusion Criteria

The exclusion criteria were as follows: (1) those with abnormal liver functions and renal insufficiency; (2) those who were in pregnancy or lactation period; (3) those with other rheumatic immune diseases such as systemic lupus erythematosus, ankylosing spondylitis, and severe osteoarthritis; (4) those with the mental disorders or patients who could not coordinate with others due to the mental retardation; (5) those with the severe diseases in vital organs such as respiration, digestion, cardio-cerebral vessels; and (6) those who were also participating in other experiments.

### 2.3. Methods

#### 2.3.1. Detection of MSUS

The color doppler ultrasound (manufacturer: Shenzhen Baisheng Medical Technology Co., Ltd.; model: CARIS) was used for examination. The patients were informed of the attention points before detection, and the detection was carried out when the patient's spirit and emotions were in a stable state. The proximal digital joints, wrist joint, carpometacarpal joint, and knee joint were scanned by conventional imaging using the model of high-frequency ultrasound. The scanning direction was consistent with the long axis of the muscle, and the patients were advised to relax the muscle during the detection. If the abnormality was detected in the above joints, the abnormal position should be examined by cross-sectional scan to compare and analyze the cross-sectional scanning images and scanning images by conventional imaging to determine the effusion and swelling of the affected joint. The specific modes of ultrasonic scan in joints were as follows: (1) The probe should be placed in the anterior segment of the shoulder joint in a horizontal position when scanning the shoulder joint. After the position in the long head of biceps tendon and the intertubercular sulcus of the femur was determined by conventional scanning, the axis of the long head of the biceps tendon was taken as the scanning direction. It should be gradually scanned from the subscapular tendon to the position of the supraspinatus, inferior gemellus muscle, and teres minor. (2) When scanning the hip joint, the ultrasound probe was placed in the parallel position of the femoral neck after the patients were in a supine position to perform the anterior scan, and the joint imaging in the femoral head and femoral neck were gradually scanned. (3) The scanning in longitudinal position and transverse position was performed when scanning the proximal finger joint and carpometacarpal joint to observe the tendon around the joint, joint surface, and joint cavity effusion in turn and the changes in morphology. (4) When scanning the knee joint, the patients were in a supine position to make them buckle the knee joint in the lower limb of the affected side, and the ultrasonic probe was placed above the apex of the patella. The cutting position in declivity was taken for scanning to record the joint cavity effusion and morphology of patients after observing the lesions in knee joint ligaments, cartilage, and synovial of the affected side.

#### 2.3.2. Semiquantitative Score

(1) Synovial proliferation. The normal range was 0 points. The periosteal proliferation was confined to the joint angle and did not exceed the connection of the highest peak in bone surface, which was 1 point. The periosteal proliferation exceeded the connection of the highest peak in bone surface, but it did not extend to the backbone as 2 points. The periosteal proliferation extended to the backbone at 3 points. (2) Bone erosion. The normal range was 0 points. The cortical bone was surface roughness without defect as 1 point, the obvious bone defect was 2 points, and the bone defect with a larger area was 3 points. (3) Joint cavity effusion. The normal range was 0 points, the paucity was 1 point, the medium was 2 points, and the mass was 3 points. (7) Intrasynovial blood signals. The normal range was 0 points. The single blood signal appeared as 1 point. The blood signals less than 50% of the synovial area were 2 points. The blood signals in more than 50% of the synovial area were 3 points.

### 2.4. Evaluation of the Oswestry Disability Index

The rating scale of the ODI [15] was used to evaluate the effect of pain on the daily activities of RA patients. There were 10 items on the scale, including the evaluation of three fields, namely, pain (degree of pain and the effect of pain on sleep), monomial function (lifting weight, sitting, standing, and walking), and individual comprehensive function (daily activity ability, sexual life, social activities, and outing). The lowest and the highest scores for each item were 0 and 5 points. The higher the score, the more serious the dysfunction of patients. 100 questionnaires were given out and recovered in this study, with an effective rate of 100%.

### 2.5. Observation Indices

The Spearman correlation analysis was used to study the relationship between the degree of illness of patients and parameters of MSUS and ODI.

### 2.6. Statistic Treatment

The experimental data were analyzed and processed by SPSS21.0, and GraphPad Prism 7 (GraphPad Software, San Diego, USA) was used to draw pictures of the data. The study data including enumeration data and measurement data were tested by *χ*^2^ and *t*-test, indicated by (n (%)) and ($\bar{x}$ ± *s*). When *P* < 0.05, the differences were considered to be statistically significant.

## 3. Results

### 3.1. Comparison of Semiquantitative Scores of MSUS in Each Group

The total semiquantitative score of MSUS in the remission group was obviously lower than that in the other three groups (*P* < 0.001). See details in Table 1.

### 3.2. Correlation between the Degree of Illness and Parameters of MSUS

The degree of illness in elderly patients with RA was positively correlated with parameters of MSUS (*r* = 0.886, *P* < 0.001). See details in Figure 1.

### 3.3. Rating Scale of the ODI in Each Group

The ODI score in the remission group was obviously lower than that in the other three groups (*P* < 0.001). See details in Table 2.

### 3.4. Correlation between the Degree of Illness and ODI

The degree of illness in elderly patients with RA was positively correlated with ODI (*r* = 0.907, *P* < 0.001). See details in Figure 2.

## 4. Discussion

The pathological changes of RA manifest as an inflammatory response of synovial joints first, and a large number of new blood vessels form with the invasiveness of inflammatory cells, thereby developing into pannus, whose presence can damage cartilage tissue and joint function. Previous studies have suggested that histopathological changes only occur when RA develops to the end stage, but subsequent studies have found that histopathological changes have occurred in the 6^th^–12^th^ week of the inflammatory response of synovial membrane, and early intervention on diagnosis and treatment can effectively organize the disease progression, thus improving the prognosis. Therefore, early diagnosis and accurate assessment of the severity of RA have a great significance in improving prognosis [16], and early diagnosis and assessment of RA are mainly by imaging examination in the clinic. Characterized by no wound, simple operation, and repeated examination, MSUS can effectively avoid the radiation injuries of CT and X-ray examination. Compared with MRI, MSUS has a lower inspection cost, and its diagnostic value has been confirmed in the diseases like traumatic superficial soft tissue injury and chronic low back pain [17]. However, in terms of the diagnosis of RA, MSUS can make use of a high-frequency probe to observe the superficial joints better, analyze the direction and velocity of blood flow by transforming into color images related to blood vessels using ultrasound, better identify the effusion and synovial proliferation in the joint cavity of patients with RA, and explore the rich blood flow signals of pannus during inflammatory activity, so as to better reflect the bone metabolic status and objectively evaluate the state of osteonecrosis in patients. Bone erosion and periosteal proliferation are the main lesions of RA, and the semiquantitative scoring system can be used to evaluate various lesions of RA in the clinic to determine the degree and location of lesions in patients [17]. Relevant literature has pointed out that MSUS can observe the tissues and organs in vivo in real time, which is suitable for displaying the morphology and interaction of muscles, tendons, bones, and joints in active, passive, or resistant motion states, and is conducive to the diagnosis of exercise-related diseases and impaction syndrome [18]. In this study, the scores were evaluated according to different grades, which were summarized as remission stage, low activity stage, middle activity stage, and high activity stage. With the increase in disease degree, the semiquantitative scores of MSUS in different groups would increase, indicating that the consistency between diagnosis of MSUS and disease degree was good. The degree of illness in elderly patients with RA was positively correlated with parameters of MSUS (*r* = 0.886, *P* < 0.001), which was consistent with the results of Zaragoza-García Oscar et al [19]. At the same time, Naqvi Atta Abbas et al. [20] showed that the DAS28 score was used to evaluate the condition of patients diagnosed with RA, and the analysis found that the semiquantitative score of MSUS increased significantly with the increase of the disease severity of RA, suggesting that the semiquantitative score of MSUS can determine the condition of RA. In addition, Sandoughi Mahnaz et al. [21] randomly selected 380 patients with RA as the research subjects. After analysis, it was found that the total score of assessment on MSUS was positively correlated with the swollen joint count and tender joint count in RA and was positively correlated with the degree of disease in patients with RA, considering that the MSUS score was closely related to the condition of RA. The above results confirmed that there was a close correlation between the parameters of MSUS and the severity of patients with RA, which is convenient to provide relevant reference data for the diagnosis and treatment of diseases.

RA is a common disease in clinics, and practical and simple assessment methods are particularly important in judging conditions, guiding treatment, observing the curative effect, and estimating prognosis [22]. The international general scales are used to evaluate the function of patients, so as to facilitate the comparison of clinical data and the development of multicountry and multicenter clinical research experiments [23]. ODI is the most commonly used scale to evaluate the dysfunction of low back pain in the world, which has been translated into Chinese by domestic scholars, with the reliability of the repeated test after Chinesization as high as 0.95, and the Chinese version is clear and easy to understand, which provides a further basis for clinical application in China [24]. The results of this study showed that the ODI score in the remission group was obviously lower than that in the other three groups, indicating that RA patients with more severe illness have a higher ODI. At the same time, the results of this study showed that the degree of illness in elderly patients with RA was positively correlated with ODI (*r* = 0.907, *P* < 0.001), which was consistent with the findings of Wang Jiawei et al [25]. The reason is that the ODI scale is fairly comprehensive, with good preciseness and professionalism in some aspects like structure, verbal expression, and content, and patients can fully understand the content of the scale in self-assessment, thus providing a good reference for the evaluation of the condition in clinic. The shortcomings of this study were as follows. First of all, the cases selected in this study were all patients in the local hospitals, with a single source of cases. Second, a sufficient sample size was not included in this study due to the limited observation time, resulting in the bias of study results. Finally, there is an inherent selection bias in a retrospective study, such as technology differences of staff in MSUS examination. Therefore, the study design should be improved, the sample size should be increased, and the relationship between the degree of illness in elderly patients with RA and parameters of MSUS and ODI, and the clinical value should be discussed in detail from multiple perspectives and aspects in the future. In summary, the preliminary conclusions obtained by this study still need to be further improved.

## Figures and Tables

**Figure 1:** Correlation between the degree of illness and parameters of MSUS.

**Figure 2:** Correlation between the degree of illness and ODI.

**Table 1:** Comparison of semiquantitative scores of MSUS in each group ($\bar{x}$ ± *s*).

Groups	*n*	Synovial proliferation	Bone erosion	Joint cavity effusion	Intrasynovial blood signals	Total score
Remission group	25	0.83 ± 0.07	0.78 ± 0.13	0.48 ± 0.09	0.59 ± 0.09	2.68 ± 0.13
Low activity group	25	2.95 ± 0.15	1.20 ± 0.18	1.08 ± 0.13	1.37 ± 0.20	6.63 ± 0.42^*∗*^
Middle activity group	25	4.11 ± 0.20	2.01 ± 0.23	2.01 ± 0.25	1.98 ± 0.33	10.03 ± 0.56^#^
High activity group	25	7.08 ± 0.70	2.15 ± 0.62	2.42 ± 0.18	2.61 ± 0.24	14.26 ± 1.24^a^

^*∗*^indicates a significant difference in total score between the low activity group and the remission group (*t* = 44.921, *P* < 0.001). ^#^indicates a significant difference in total score between the middle activity group and the remission group (*t* = 63.925, *P* < 0.001). ^a^indicates a significant difference in total score between the high activity group and the remission group (*t* = 46.439, *P* < 0.001).

**Table 2:** Rating scale of ODI in each group ($\bar{x}$ ± *s*).

Groups	N	ODI score
Remission group	25	8.32 ± 2.13
Low activity group	25	15.16 ± 1.35^*∗*^
Middle activity group	25	20.95 ± 1.69^#^
High activity group	25	28.64 ± 1.81^a^

^*∗*^indicates a significant difference in ODI score between the low activity group and the remission group (*t* = 13.471, *P* < 0.001). ^#^indicates a significant difference in ODI score between the middle activity group and the remission group (*t* = 23.092, *P* < 0.001). ^a^ indicates a significant difference in the ODI score between the high activity group and the remission group (*t* = 36.151, *P* < 0.001).

## Data Availability

The data used to support the findings of this study are available upon reasonable request from the corresponding author.
